RETRACTED

# Harnessing TRAIL-Induced Apoptosis Pathway for Cancer Immunotherapy and Associated Challenges

**DOI:** 10.3389/fimmu.2021.699746

**Published:** 2021-08-20

**Authors:** Ehsan Razeghian, Wanich Suksatan, Heshu Sulaiman Rahman, Dmitry O. Bokov, Walid Kamal Abdelbasset, Ali Hassanzadeh, Faroogh Marofi, Mahboubeh Yazdanifar, Mostafa Jarahian

**Affiliations:** ^1^Human Genetics Division, Medical Biotechnology Department, National Institute of Genetics Engineering and Biotechnology (NIGEB), Tehran, Iran; ^2^Faculty of Nursing, HRH Princess Chulabhorn College of Medical Science, Chulabhorn Royal Academy, Bangkok, Thailand; ^3^Department of Physiology, College of Medicine, University of Suleimanyah, Suleimanyah, Iraq; ^4^Department of Medical Laboratory Sciences, Komar University of Science and Technology, Sulaimaniyah, Iraq; ^5^Institute of Pharmacy, Sechenov First Moscow State Medical University, Moscow, Russia; ^6^Laboratory of Food Chemistry, Federal Research Center of Nutrition, Biotechnology and Food Safety, Moscow, Russia; ^7^Department of Health and Rehabilitation Sciences, College of Applied Medical Sciences, Prince Sattam bin Abdulaziz University, Al Kharj, Saudi Arabia; ^8^Department of Physical Therapy, Kasr Al-Aini Hospital, Cairo University, Giza, Egypt; ^9^Department of Applied Cell Sciences, School of Advanced Technologies in Medicine, Tehran University of Medical Sciences, Tehran, Iran; ^10^Immunology Research Center (IRC), Tabriz University of Medical Sciences, Tabriz, Iran; ^11^Stem Cell Transplantation and Regenerative Medicine, Department of Pediatrics, Stanford University School of Medicine, Palo Alto, CA, United States; ^12^Toxicology and Chemotherapy Unit (G401), German Cancer Research Center, Heidelberg, Germany

**Keywords:** tumor necrosis factor-related apoptosis-inducing ligand, mesenchymal stem/stromal cells, resistance, nanoparticles, combination therapy

## Abstract

The immune cytokine tumor necrosis factor-related apoptosis-inducing ligand (TRAIL) has attracted rapidly evolving attention as a cancer treatment modality because of its competence to selectively eliminate tumor cells without instigating toxicity *in vivo*. TRAIL has revealed encouraging promise in preclinical reports in animal models as a cancer treatment option; however, the foremost constraint of the TRAIL therapy is the advancement of TRAIL resistance through a myriad of mechanisms in tumor cells. Investigations have documented that improvement of the expression of anti-apoptotic proteins and survival or proliferation involved signaling pathways concurrently suppressing the expression of pro-apoptotic proteins along with down-regulation of expression of TRAILR1 and TRAILR2, also known as death receptor 4 and 5 (DR4/5) are reliable for tumor cells resistance to TRAIL. Therefore, it seems that the development of a therapeutic approach for overcoming TRAIL resistance is of paramount importance. Studies currently have shown that combined treatment with anti-tumor agents, ranging from synthetic agents to natural products, and TRAIL could result in induction of apoptosis in TRAIL-resistant cells. Also, human mesenchymal stem/stromal cells (MSCs) engineered to generate and deliver TRAIL can provide both targeted and continued delivery of this apoptosis-inducing cytokine. Similarly, nanoparticle (NPs)-based TRAIL delivery offers novel platforms to defeat barricades to TRAIL therapeutic delivery. In the current review, we will focus on underlying mechanisms contributed to inducing resistance to TRAIL in tumor cells, and also discuss recent findings concerning the therapeutic efficacy of combined treatment of TRAIL with other antitumor compounds, and also TRAIL-delivery using human MSCs and NPs to overcome tumor cells resistance to TRAIL.

RETRACTED

## Introduction

The tumor necrosis factor-related apoptosis-inducing ligand (TRAIL) belongs to the group of chemotherapeutic ingredients, which specifically affects various tumor cells without targeting the normal cells (1). It has been evidenced that due to lower expression of TRAIL receptors on the surface of normal cells, theses cell are inherently resistant to TRAIL-induced apoptosis (2). However, deregulation of various signaling molecules and pathways, such as Janus kinase (JAK) and P53, results eventually in up-regulation of TRAIL-receptors expression, leading to tumor cells elimination (3–5). The well-known therapeutic competence of TRAIL has robustly relied on the expression of its receptors in a variety of cells and tissues, ranging from lymphocytes to spleen, thymus, ovary, prostate, colon, intestine, and placenta; while the expression of identified receptors for other ligands of the TNF family are commonly restricted and transient (6, 7). Though the Fas/FasL and TNFα/TNFR1 are identified to stimulate the oncogenic NF-κB pathway, TRAIL elicits a weak influence on NF-κB stimulation, reflecting its superior safety as a therapeutic agent (8). Interestingly, TRAIL also contributes to the natural killer (NK) cell-induced immunosurveillance toward metastatic cancer cells, describing TRAIL as a favorable and effective anticancer molecule for clinical application. TRAIL as a cytokine is frequently expressed by immune cells and plays a prominent role in T-cell homeostasis and NK or T-cell mediated elimination of malignant cells (9, 10). This cytokine is considered a type II transmembrane protein containing an extracellular domain, which generates its biologically active soluble form upon cleavage.

RETRACTED

In the present review, we will describe TRAIL signaling and its regulation, as well as known mechanisms that contributed to cancer cell resistance to TRAIL therapy, and more importantly, will investigate the current approaches that resistance, ranging from combination therapy (using TRAIL along with other anti-tumor agents) to TRAIL targeted delivery by nanoparticles (NPs) and stem cells (SCs).

### TRAIL Signaling and Its Regulation

TRAIL interacts with two agonistic receptors, including TRAIL-R1 (DR4) and TRAIL-R2 (DR5), and three antagonistic receptors, encompassing TRAIL-R3 (DcR1), TRAIL-R4 (DcR2), and soluble receptor osteoprotegerin (OPG) (**Figure 1**) (2). TRAIL-R1 and TRAIL-R2 expression is typically adjusted through p53, and TRAIL-R2 gene promoter includes a p53 receptive component.

**Figure 1:** The recognized receptors for TRAIL. TRAIL connects with two agonistic receptors, termed TRAIL-R1 (DR4) and TRAIL-R2 (DR5), and three antagonistic receptors, termed TRAIL-R3 (DcR1), TRAIL-R4 (DcR2) as well as a soluble receptor, known as osteoprotegerin (OPG). TRAIL, Tumor necrosis factor-related apoptosis inducing ligand.

In addition to the stimulation of apoptosis in TRAIL-sensitive cells, TRAIL-R1 and TRAIL-R2 can elicit the survival involved signaling axis in malignant cells, thus hindering cell death following treatment with TRAIL (11). TRAIL interaction with its receptors can result in the activation of either extrinsic or intrinsic apoptosis pathways in tumor cells, in which the interrelation between these pathways is attributed by the truncation of the BH3-domain interacting protein (Bid). Mechanistically, TRAIL connecting to its two death receptors, DR4 and DR5, leads to the triggering of the extrinsic pathway, which continues with trimerization of receptors and formation of the death-inducing signaling complex (DISC) (12, 13). Fas-associated death domain protein (FADD), but not Fas, are recruited to the DISC, and interrelates with the death domains (DD) in the cytoplasmic region of DR4 and DR5, enabling the translocation and succeeding activation of procaspase-8/10 by communication of their respective death effector domains (DED) (14). In the intrinsic pathway, caspase-8 activation supports cleavage of pro-apoptotic protein Bid, and then the truncated Bid interrelates with other well-known pro-apoptotic proteins, Bax and Bak. This interaction facilitates Bax and Bak oligomerization in the mitochondrial membrane, supporting a modification in mitochondrial membrane potential (ΔΨm) and eventually secretion of cytochrome (cyt) c and Smac/Diablo (15, 16) (**Figure 2**). The conventional suggested model for DISC assembly and structure implies that FADD is substoichiometric and procaspase-8 is recruited by both contacting with FADD and also interrelating with itself.

RETRACTED

**Figure 2:** The mechanism of TRAIL-induced apoptosis in tumor cells. TRAIL connecting to DR4 and DR5 stimulates apoptosis in both the extrinsic and intrinsic pathways following trimerization of receptors and FADD translocation and activation. However, various anti-apoptotic proteins, including c-FLIP, XIAP, Mcl-1, survivin, Bcl-2, and Bcl-xL can negatively regulate apoptosis pathways. TRAIL, Tumor necrosis factor-related apoptosis-inducing ligand; DRs, Death receptors; FADD, FAS-associating death domain-containing protein; c-FLIP, Cellular FLICE (FADD-like IL-1b-converting enzyme)-inhibitory protein; Bcl-2, B-cell lymphoma-2; Bcl-xl, B-cell lymphoma-extra large; Mcl-1, Myeloid-cell leukemia 1; XIAP, X-linked inhibitor of apoptosis; Bax, Bcl-2 associated X; Bak, Bcl-2 homologous antagonist/killer; Bid, BH3-interacting domain death agonist.

This apoptotic pathway is tightly regulated. At the DISC, caspase-8/10 stimulation can be suppressed by anti-apoptotic protein cellular FLICE-like inhibitory protein (c-FLIP) (17). On the other hand, anti-apoptotic proteins, X-linked inhibitor of apoptosis protein (XIAP), and survivin can trigger straight suppression of the effector caspases activity, whereas the suppressive activity of XIAP on caspases is modified strongly by at least two XIAP-interacting proteins, XAF1 and Smac/Diablo (18, 19). Moreover, regardless of the two most important members of the anti-apoptotic Bcl-2 family protein, Bcl-2 or Bcl-xL (20), which their activities robustly inhibits Bax-mediated apoptosis, Mcl-1 as another Bcl-2 family protein plays a pivotal role in the regulation of apoptosis and also upholding cell survival by interrupting some axis which supports the release of cytochrome c from mitochondria (21, 22).

Pre-clinical investigations have revealed that the utility of the soluble (s) and also full-length (FL) form of TRAIL in animal models could inhibit the proliferation of TRAIL-sensitive human tumor xenografts without any serious systemic toxicity, sustaining the potent application of TRAIL *in vivo* (23–25). Nonetheless, the chief restriction of TRAIL therapy is the progress of TRAIL resistance by a variety of mechanisms in target cells (26, 27). Based on the literature, up-regulating anti-apoptotic proteins and survival or proliferation involved signaling axis concomitant with down-regulating pro-apoptotic proteins, as well as DR4/5 expression and activation seem to play a crucial role in cancer cells resistance to TRAIL (28, 29). Hence, for improvement of the TRAIL elicited anti-tumor effects, combined use of TRAIL with various TRAIL sensitizing components (e.g., synthetic agents and natural products) has represented pronounced therapeutic outcomes. Further, the use of NPs and stem cells, in particular, human mesenchymal stem/stromal cells (MSCs), as TRAIL delivery vehicles has currently attracted rapidly evolving attention (30–32).

RETRACTED

## Mechanisms of Cancer Resistances to Trail

### Anti-Apoptotic Proteins in TRAIL Resistance

In 1998, Griffith et al. showed that presence or the absence of intracellular apoptosis inhibitors could mediate resistance or sensitivity to TRAIL-induced apoptosis in melanoma cell lines (33). After that, in 1999, Tepper and Seldin described that there is a direct association between expression levels of the anti-apoptotic protein c-FLIP and resistance to apoptosis-inducing molecules, such as Fas, in a cancer cell line *in vitro*. They found that the relative levels of caspase-8 and c-FLIP act as a determinant factor affecting susceptibility to Fas -induced apoptosis in Burkitt’s lymphoma (BL) (34). Similarly, another report suggested that tumor cell evasion from T cell immunosurveillance may rely on the c-FLIP expression in human melanomas *in vivo*. Correspondingly, c-FLIP overexpression resulted in marked resistance to Fas -induced apoptosis in tumor cells *in vitro* (35). Besides, c-FLIP averts caspase-8 cleavage in breast carcinoma cell line T47D and negatively regulates cell death in T47D cells (36). In a similar pattern, it has been found that c-FLIP is typically expressed in human hepatocellular carcinomas (HCCs) cells at a higher level than in non-tumor liver tissues. As well, c-FLIP down-regulation exerted by cFLIP antisense oligodeoxynucleotides made HCCs susceptible to TRAIL-, and - Fas mediated apoptosis, and conversely, its over-expression intensified cells resistance to apoptosis-inducing agents, more importantly *via* inhibition of caspase-8 activation concurrently promoting nuclear factor (NF)-κB activation (37). These results indicate that c-FLIP participates in cell survival by both blocking death-receptor-mediated apoptosis and adjusting NF-κB activation in human HCCs (37).

Likewise, Bcl-xL, a cellular inhibitor of apoptosis 2 (cIAP2) and survivin down-regulating following silencing of zinc finger protein SNAIL, which in turn, sustained HCC cells susceptibility to TRAIL-mediated apoptosis signified the chief role of the anti-apoptotic proteins in the resistance process of tumor cells to TRAIL (38). Besides, investigation of the TRAIL effects on non-small cell lung cancer (NSCLC) cell line, NCI-H460, verified tumor cell’s sensitivity to TRAIL, while Bcl-2 overexpression supported a highly TRAIL-resistant phenotype, and thereby evidenced the importance of the mitochondrial pathway in stimulating TRAIL-induced apoptosis. Interestingly, Bcl-2 overexpression largely suppressed the final cleavage in caspase-8 and also caspase-3; on the other hand, XIAP knockdown led to the improvement of the cellular levels of cleaved caspase-3 upon treatment with TRAIL (39). Cingöz and his coworkers showed that TRAIL-mediated apoptosis in glioblastoma (GBM) cell lines can be promoted following combination therapy with proteasome inhibitor bortezomib and TRAIL, evidently by down-regulating Bcl-2 or Bcl-xL, suggesting a role for these anti-apoptotic proteins in inducing resistance to apoptosis-inducing cytokines, in particular, TRAIL (40). Moreover, analysis of the apoptosis process induced by TRAIL in human colon cancer cell line SW620 revealed that although caspase-8 activation and subsequent tBid formation was triggered in tumor cells upon treatment with TRAIL, up-regulating Bcl-2, Bcl-xL and Mcl-1 blocked TRAIL-mediated apoptosis in treated tumor cells (41). Conversely, Lippa et al. found that the steady blocking of the XIAP in human colon carcinoma cell line Colo320 subcutaneous tumors led to the delayed tumor growth and also supported susceptibility to TRAIL exerted anti-tumor functions *in vivo* (42). Considering other studies, up-regulating Mcl-1 in melanoma cells is proposed to boost tumor cells resistance to TRAIL-mediated apoptosis, while combination therapy with Mcl‐1‐selective inhibitor S63845 with TRAIL improved robust apoptosis in TRAIL-resistant melanoma cells, and thereby confirmed the influential role of the Mcl-1 in determining the cell responses to TRAIL (21).

RETRACTED

### Pro-Apoptotic Proteins in TRAIL Resistance

A large number of studies suggest that DRs-mediated apoptosis in tumor cells may arise from inducing pro-apoptotic proteins, such as Bax. In 2002, LeBlanc et al. found that Bax-deficient human colon carcinoma cells show remarkable resistance to death-receptor ligands, while Bax-expressing sister clones were susceptible. They suggested that although Bax is unessential for apical death-receptor signaling actions like caspase-8 induction, this pro-apoptotic protein largely contributes to mitochondrial changes and downstream caspase induction (43). Likewise, other reports revealed that Bax null tumor cells were resistant to TRAIL-induced apoptosis; however, Bax deficiency had no impact on TRAIL-induced caspase-8 induction and following cleavage of Bid. Given that Bax deficiency supports imperfect caspase-3 processing due to the inhibition by XIAP, observations indicated that secretion of Smac/Diablo from mitochondria by the TRAIL-caspase-8-tBid-Bax cascade is essential for removing the negative effect of the XIAP on apoptosis. Therefore, Deng et al. suggested that Bax-dependent secretion of Smac/Diablo, but not cytochrome c, from mitochondria participate in TRAIL-induced apoptosis (44). Further, tumor stem cells derived from patients with the most malignant primary brain tumor, medulloblastoma (MB), demonstrated robust resistance to TRAIL-induced apoptosis. The analysis showed that several mechanisms, in particular, down-regulating Bax in tumor stem cells were responsible for the defect in TRAIL-induced apoptosis (45). In this regard, other studies have shown that despite the Bak expression, Bax-deficient cells demonstrated resistance to TRAIL-induced apoptosis. Indeed, Bax dependency of TRAIL-elicited cell death is determined through Mcl-1 but not Bcl-xL, whereas silencing of Mcl-1 but not Bcl-xL could defeat resistance to TRAIL in Bax-deficient cells, and also facilitate Bak inducing by TRAIL (46).

Resistance to TRAIL can be caused by activation of protein kinase C-epsilon (PKCepsilon) which inhibits caspase-8 and -9 activation as well as hindering cytochrome c secretion from mitochondria, as shown in MCF-7 breast cancer cells (47). The PKCepsilon functions result in improvement in Bcl-2 expression, and also reduction in Bid expression without any effect on Bax, and thus implying that it arbitrates TRAIL resistance through both Bcl-2 and Bid in breast cancer cells (47).

Studies have shown that resistance of the oral squamous cell carcinoma (OSCC) to TRAIL-induced apoptosis is mediated by RANK ligand (RANKL) activation and subsequent blocking of pro-apoptotic proteins Bad and Bax, highlighting the importance of the pro-apoptotic proteins in TRAIL-induced OSCC tumor cell apoptosis (48). Moreover, resistance to TRAIL in TRAIL-resistant SW480 cells is mediated by up-regulating miR-20a. Silencing miR-20a and subsequent Bid activation renders SW40 cells sensitive to TRAIL-induced apoptosis which supports the central biological role of pro-apoptotic proteins in determining the tumor cell response to TRAIL (49). Consistently, Lee et al. described that although combination therapy with TRAIL and other compounds could make human colon cancer HCT116 cell line susceptible to TRAIL, Bax-deficient cells but not Bak-deficient cells, restored their resistance to TRAIL (50). In sum, these findings imply that the TRAIL-induced apoptosis is closely linked to Bax-mediated mitochondria-dependent pathway.

### Main Survival-Involved Signaling Axis in TRAIL Resistance

#### NF-κB

Previous studies have supported that activation of NF-κB by Epstein-Barr virus (EBV) infection largely participates in resistance of BL cell lines to TRAIL-induced apoptosis, and consequently, application of NF-κB inhibitors may be valuable for defeating BL cells resistance to TRAIL (**Figure 3**) (36). Similarly, NF-κB activation is responsible for the resistance of wild-type (WT) leukemia cell line HL60 cells, to TRAIL, as shown by investigating TRAIL-resistant HL60 subclones (51). Also, Beyer et al. showed that NSCLC-acquired resistance to TRAIL was arbitrated by NF-κB up-regulation; however, they also observed that p53-independent apoptosis by attenuating NF-κB expression and concurrently suppressing Bcl-2 and Bcl-xL activities in NSCLC, may be responsible for TRAIL-induced apoptosis upon combination therapy with TRAIL and other anti-tumor agents (52). Further, NF-κB activation as a downstream target of the glycogen synthase kinase-3β (GSK-3β) activating in lung cancer cells has been presented as another possible mechanism involved in inducing resistance to TRAIL (53). Interestingly, there is some evidence indicating that TRAIL interrelation with DcR2 may result in NF-κB activation in large granular lymphocyte (LGL) leukemia. Regardless of detecting up-regulated TRAIL messenger RNA and protein expression in LGL leukemia cells, studies have shown that DcR2 is the principal TRAIL receptor in LGL leukemia cells, and also evinced that TRAIL-elicited activation of DcR2 caused augmented NF-κB activation in leukemic LGL cells (54). Moreover, expression of a set of NF-κB-regulated microRNAs, such as miR-21, miR-30c, and miR-100, which affect tumor-suppressor genes, are suggested to be involved in acquiring resistance to TRAIL in lung cancer cells (55). Likewise, NF-κB contributes to supporting resistance to TRAIL in melanoma (56), bladder cancers (57), and also glioblastoma (58).

RETRACTED

**Figure 3:** The bortezomib-mediated process involved in inducing TRAIL-mediated apoptosis in TRAIL-resistant tumor cells. The proteasome inhibitor bortezomib prohibits NF-κB activation and consequently down-regulates anti-apoptotic protein expression in target cells, sensitizing TRAIL-resistant tumor cells to TRAIL-induced apoptosis. TRAIL, Tumor necrosis factor-related apoptosis-inducing ligand; NF -κB, Nuclear factor-kappa B; IκB, Inhibitor kappa B.

#### Akt

In addition to the NF-κB, Akt activation induces tumor cell resistance to the apoptosis-inducing agents (e.g., TRAIL). A myriad of tumor cells such as prostate cancer cells, express active Akt because of the loss of lipid phosphatase PTEN gene, a prominent inhibitor of phosphatidylinositol 3-kinase (PI3K) pathway (**Figure 4**). Thereby, tumor cell lines that express the high level of Akt marked resistance to apoptosis by TRAIL. In contrast, inhibiting Akt activities by PI3K inhibitors, wortmannin and LY294002, abrogated cellular resistance to TRAIL. Importantly, transfection of the constitutively active Akt into tumor cells with low Akt activity could result in reinforced Akt activity and then modified TRAIL-induced apoptosis (59). Given that Akt is negatively modified by the tumor suppressor PTEN, researchers evaluated tumor cell’s sensitivity to TRAIL in PTEN knockdown murine prostate epithelial cells. Unsurprisingly, they found that PTEN−/− cells were more resistant than PTEN+/+ to TRAIL-induced apoptosis, and also overexpression of a mutant PTEN diminished TRAIL resistance in PTEN+/+ cells, presenting the pivotal role of PTEN in TRAIL sensitivity (60). Also, it has been found that liver cancer stem cells (LCSCs) resistance to TRAIL is sustained by miR-21-3p overexpression, which acts as an inhibitor of PTEN and thereby positively regulates Akt activation in xenografts nude mice (61). Also, Akt up-regulation is deemed to negatively modify apoptotic proteins during early steps of TRAIL-induced apoptosis in colorectal carcinoma (62), lung cancer (63), glioma (64), neuroblastoma (65), HCC (66, 67), and gastric cancers (68).

**Figure 4:** The PTEN important roles in the regulation of cell response to TRAIL. Downregulation of PTEN results in unregulated activation of the PI3K/Akt pathway, which in turn, leads to the tumor cell’s resistance to TRAIL. Nonetheless, PTEN up-regulating using therapeutic agents plus TRAIL may support TRAIL-induced apoptosis in TRAIL-resistant cells. TTRAIL, umor necrosis factor-related apoptosis-inducing ligand; PTEN, Phosphatase and tensin homolog; NF -kB, Nuclear actor-kappa B; mTOR, Mechanistic target of rapamycin; PI3K/AKT, Phosphatidylinositol 3-kinase; IKK, IkB kinase; FOXO, forkhead box transcription factors; Bad, Bcl2 associated agonist of cell death; RHEB, Ras homolog enriched in brain; S6K, S6 kinase; eIF4E, Eukaryotic translation initiation factor 4E.

#### ERK

ERK is known as another prominent protein capable of potently suppressing TRAIL-induced release of Smac/Diablo in melanoma cells, and thereby diminishing their sensitivity to TRAIL. Conversely, blocking ERK signaling using MEK inhibitor U0126 or a dominant-negative mutant of MKK1 could sustain melanoma cells susceptible to TRAIL-induced apoptosis (69). ERK signaling axis is suggested to protect melanoma cells toward TRAIL-induced apoptosis by suppressing Bax activation, which in turn, could reduce TRAIL-mediated secretion of Smac/Diablo and activation of apoptosis (69). Besides, studies on TRAIL-resistant sub-population of the HCC cell line LH86 revealed that Musashi RNA binding protein 1 (Msi1) expression which enables ERK activation was responsible for inducing resistance to TRAIL. Meanwhile, overexpression of Msi1 diminished the sensitivity of HCC cells to TRAIL both *in vitro* and *in vivo*, while siRNA-mediated exhaustion of ERK defeated TRAIL resistance (70). Furthermore, assessment of the underlying mechanisms that contribute to acquired resistance to TRAIL in TRAIL-resistant human ovarian cancer cell lines (SKOV-3ip1 and A2780) showed that DR4/5-indued signaling following their bindings to TRAIL undesirably elicits induction of pro-survival factors such as NF-κB, Akt, and ERK(1/2), potentiating tumor cells resistance to TRAIL-mediated apoptosis (71). Also, heterogeneous nuclear ribonucleoprotein K (hnRNPK) activation resulting from ERK up-regulating in lung adenocarcinoma H1299 cells is closely related to hnRNPK-mediated TRAIL resistance in H1299 cells. Accordingly, ERK1/2 facilitates the cytoplasmic accumulation of hnRNPK and therefore abolishes TRAIL-induced apoptosis by positive regulation of XIAP in H1299 cells (72). Besides, recent findings have shown that growth arrest and DNA damage-inducible protein 34 (GADD34) constrains TRAIL-induced HCC cell apoptosis by ERK-arbitrated stabilization of anti-apoptotic protein Mcl-1 and suppression of its degradation (72, 73). Furthermore, ERK activation may provoke acquired TRAIL resistance in cancers of the breast (74), colon (75), gastric (76), cervical (77), renal carcinoma (78), and also neuroblastoma (79).

RETRACTED

### Death Receptors and Resistance to TRAIL

Studies on TRAIL-resistant SW480 human colon adenocarcinoma cells revealed that although the total cellular DR4 proteins are commonly identified in TRAIL-sensitive and TRAIL-resistant clones; the resistant cells virtually show lower rates of DR4 on the cell surface. Further, exogenous DR4 and DR5 may not be properly transported to the TRAIL-resistant cell surface; however, pre-exposure with tunicamycin which enables DR4/5 expression on cell surface, re-sensitizes resistant cells to TRAIL. These findings imply that resistance to TRAIL can be prohibited by adjusting the transport of death receptors to the cell surface (80). Other investigations on human pancreatic cancer cell lines PANC-1 and BxPC-3 showed that treatment with TRAIL reduced the expression of DR4 and pointedly improved DCR1/2 expression, leading to inhibition of TRAIL-induced apoptosis, while OPG levels persisted unaffected. Interestingly, co-stimulation with TRAIL and lipopolysaccharides (LPS) more obviously promoted the variations in TRAIL-receptor-expression sponsoring apoptosis resistance due to the recognized effects of LPS on TLR-4 activation (52). On the other hand, CRISPR/Cas9 mediated silencing of DR5 suppressed bortezomib-mediated re-sensitization of glioblastoma cell lines to TRAIL-induced apoptosis, representing its significant role in determining cell response to TRAIL (40). Furthermore, it has been suggested that DCR2 could shape a heteromeric complex with the DR5 and consequently diminish caspase-8 activation and apoptosis in human cervical cancer HeLa cells. Correspondingly, ectopic expression of DCR2 in HeLa cells could trigger morphological variations along with improved cell proliferation *in vitro* as well as tumor growth *in vivo*. These findings have signified that DCR2 up-regulating leads to the activation of signaling pathways enabling cell survival and proliferation in HeLa cells (26). Moreover, Zhang et al. have suggested that loss of cell surface expression of DR4 or DR5 is reliable for attenuated sensitivity to TRAIL in human breast cancer cells. They also found that TRAIL resistance developed in the lack of DR4/5 on cell surface regardless of changes in Bcl-2 family proteins or caspases.

RETRACTED

Importantly, reserving endocytosis using pharmacologic inhibitors or interruption of clathrin-dependent endocytosis signaling molecules facilitated DR4/5 cell surface expression and then made resistant cells susceptible to TRAIL-induced apoptosis (81). In this regard, other studies presented that DR5 up-regulating upon combination therapy with TRAIL and paxilline was responsible for sensitizing TRAIL-resistance glioma cell to TRAIL-induced apoptosis mediated by a C/EBP homologous protein (CHOP)/GADD153-arbitrated process (**Figure 5**) (82). This theory declares that activating the CHOP/GADD153 axis upon treatment of TRAIL-resistant cells with various therapeutic agents may result in up-regulation of DR4/5, and consequently elicits ER stress-mediated apoptosis in these cells (82). Regardless of the central role of DR4 during TRAIL-mediated apoptosis of tumor cells, there is some proof suggesting that DR4-C626G and -A1322G polymorphisms could be considered as the molecular risk factors for non-Hodgkin lymphoma (NHL) in human (83).

**Figure 5:** The CHOP-mediated up-regulation of DR5. The ER stress stimulates the induction of PERK, which supports phosphorylation of eIF2α, and thereby results in stimulation of translation of ATF4. Then, ATF4- ATF3- CHOP signaling pathway is elicited and contributes to the up-regulating DR5 expression, facilitating tumor cells-sensitivity to TRAIL. TRAIL, Tumor necrosis factor-related apoptosis-inducing ligand, CHOP, C/EBP homologous protein; PERK, Protein kinase R-like ER kinase; eIF2α, Eukaryotic translation initiation factor 2α; ATF3/4, Activating transcription factor 3/4; ER Stress, Endoplasmic reticulum stress; DISC, Activation of death-inducing signaling complex.

RETRACTED

## Overcoming Trail Resistance Using Combination Therapy

### Synthetic Agents

As described earlier, TRAIL is suggested as an encouraging anti-cancer modality; however, many cancers are or become inherently resistant to TRAIL. Nonetheless, combination treatment can defeat TRAIL resistance and improve TRAIL-induced apoptosis in TRAIL-resistant tumor cells. Recently, combined treatment of histone deacetylase inhibitors (HDACi’s) and TRAIL have demonstrated marked capability to overcome TRAIL resistance in human cancers. TRAIL-induced apoptosis was chiefly promoted in colon cancer WiDr cells by pre-exposure to Entinostat, an HDAC1, 2, and 3 inhibitors, and in colon cancer DLD-1 cells by RGFP966, an HDAC3-specific inhibitor, or PCI34051, an HDAC8-specific inhibitor. Analysis indicated that RGFP966 and PCI34051 could stimulate DR4 expression on DLD-1 cells, while RGFP966 elicited more DR5 expression on WiDr cells, representing a dissimilar role for DR4 or DR5 in these interventions (84). Similarly, Entinostat could induce apoptosis in TRAIL-resistant melanoma following combination therapy with TRAIL by up-regulating DR4, DR5, and procaspase 8 expressions, and concurrently c-FLIP downregulating in tumor cells. Meanwhile, intensified expression of ectopic c-FLIP could negatively modify the cooperative apoptosis stimulation by the combination of entinostat and TRAIL (85). Likewise, combined treatment of TRAIL and HDACi vorinostat (suberanilohydroxamic acid, SAHA) in multiple myeloma (MM) (86), and sarcoma (87), and also HDACi valproic acid (VPA) in anaplastic thyroid carcinoma (ATC) (88), and head and neck cancer (HNC) (88) could defeat tumor cells resistance to TRAIL-induced apoptosis.

Various chemotherapeutic drugs such as 5-fluorouracil (5-FU), mitomycin, and calpain inhibitor I, an NFκB inhibitor, can make TRAIL-resistant DLD1 colon cancer cells susceptible to TRAIL-induced apoptosis. Combination therapy with TRAIL and 5-FU improved tumor inhibition *in vivo* in nude mice bearing subcutaneous tumors. While combination therapy with TRAIL and 5-FU or mitomycin caused boosted caspase-3 stimulating, the combination treatment of TRAIL and calpain inhibitor I led to improved caspase-8 and caspase-3 stimulation. Further, mitomycin but not 5-FU or calpain inhibitor I triggered pro-apoptotic protein Bax expression in TRAIL-resistant DLD1 cells (89). Also, TRAIL plus 5-FU showed remarkable cytotoxicity against TRAIL-resistant renal cell carcinoma (RCC) Caki-1 cells, and also freshly derived RCC cells from patients. Molecular studies revealed that treatment of Caki-1 cells with 5-FU supported p53 and Bax, but not Bcl-2 expression. On the other hand, treatment of Caki-1 cells with TRAIL reduced the expression of thymidylate synthase (TS) and dihydropyrimidine dehydrogenase (DPD) modestly and improved the expression of orotate phosphoribosyl transferase (OPRT) (90). Thereby, these observations verified the potential utility of combination treatment with TRAIL and 5-FU for treating TRAIL/5-FU-resistant cancer cells. Besides, cisplatin presented a synergistic impact on TRAIL-induced apoptosis in HCC cell lines mainly mediated by DR4 up-regulating. Respecting that, blocking NF-κB by specific inhibitor had no significant impact on TRAIL-induced apoptosis in HCC cells, which could indicate that NF-κB activities may not contribute to the TRAIL resistance of HCC cells (91).

RETRACTED

Furthermore, cisplatin can induce TRAIL apoptotic pathway in glioblastoma cells neurospheres by DR5 up-regulation and c-FLIP downregulation (92), and also in ovarian cancer SKOV-3 and TOV-21G cells through up-regulating Bax and caspase 3 expression and down-regulating Bcl-2 expression (93). Moreover, for enhancing the efficacy of TRAIL receptor agonists, the proteasome inhibitor bortezomib is considered one of the most effective sensitizers. For example, combined treatment with TRAIL and bortezomib supported robust synergistic response with heightened activation of caspases-8, -9, and -3, and reinforced Annexin V-binding cell fractions in TRAIL-resistant SNU-216 gastric cancer cells. Although bortezomib improved DR5 expression, DR5 silencing considerably recovered cell viability. Moreover, bortezomib reduced phosphorylation of ERK1/2, but improved JNK phosphorylation, and also bortezomib-mediated DR5 upregulation was blocked only by suppressing activation of ERK1/2 but not JNK in gastric cancer cells (94). Moreover, bortezomib could restore TRAIL-mediated apoptosis in MM cell lines, RPMI 8226 and U266, by reducing c-FLIP protein expression concomitantly enhancing DR4 and DR5 expression (95) in HPV-positive head and neck cancer (HNC) cells by ameliorating activation of caspase-8, -9, and -3, improving membrane expression of DR5, cytochrome c release, and inducing G2/M arrest (96), and also in HCC cells by inhibition of the PI3K/Akt pathway (97). Finally, it has been suggested that gemcitabine plus TRAIL could promote the responsiveness of pancreatic cancer cells to treatment with TRAIL (98).

A list of synthetic agents which recently have been applied to sensitize tumor cells to TRAIL-induced apoptosis has been cited in **Table 1**.

**Table 1:** Combination therapy with synthetic agents and TRAIL for improving TRAIL-mediated apoptosis in TRAIL-resistance cells.

Agent	Cancer	Results	Ref
**Entinostat**	Colon cancer	Up-regulation of DR4/5 in DLD-1 and WiDr cells (*in vitro*)	(84)
**Entinostat**	Melanoma	Up-regulation of DR4/5 and activation of caspase 8 (*in vitro*)	(85)
**SAHA**	MM	Induction of caspase-8 and -9 activation in OPM-2, RPMI 8226, NCI-H929, U266, and JJN-3 cells (*in vitro*)	(86)
**SAHA**	Sarcoma	Attenuating mitochondrial membrane potential and caspase-3, -6, and -7 activation, and PARP cleavage in MES-SA and ESS-1 cells (*in vitro*)	(87)
**VPA**	ATC	Activation of JNK and the phosphorylation of FADD and c-Jun, and induction of caspase-3, and -8 activation in ARO cells (*in vitro*)	(88)
**VPA**	HNC	HDAC4 degradation (*in vitro*)	(88)
**5-FU**	Colon cancer	Induction of caspase 3 activation and Bax expression in DLD-1 cells (*in vitro*)	(89)
**5-FU**	RCC	Up-regulating p53 and Bax expression in Caki-1 cells (*in vitro*)	(90)
**Cis-platin**	HCC	Up-regulating DR4 (*in vitro*)	(91)
**Cis-platin**	Glioblastoma	Up-regulation of DR5 and down-regulation of c-FLIP in glioblastoma-derived stem cells (*in vitro*)	(92)
**Cis-platin**	Ovarian cancers	Up-regulating caspase-8 and DR5 expression in SKOV-3 and TOV-21G cells (*in vitro*)	(93)
**Bortezomib**	Gastric cancer	ERK1/2 activation resulted in DR5 up-regulation, and activation of caspases-8, -9, and -3 in SNU-216 cells (*in vitro*)	(94)
**Bortezomib**	MM	Up-regulating DR5 (*in vitro*)	(99)
**Doxorubicin**	Breast cancer	DR5 activating (*in vitro* and *in vivo*)	(100)
**Gemcitabine**	Pancreatic cancer	Elevating the expression of 4E-BP1 (*in vitro*)	(98)
**Paxiline**	Glioma	Down-regulating c-FLIP, an survivin expression, and up-regulating CHOP mediated DR5 expression in U251MG cells (*in vitro*)	(82)
**SHetA2**	Lung cancer	Down-regulating c-FLIP, and up-regulating DR5 (*in vitro*)	(101)
**Actinomycin D**	Prostate cancer	Down‐regulation of XIAP, c-FLIP, Bcl-2, and up-regulation of DR4/5 in CL‐1, DU‐145, and PC‐3 cells (*in vitro*)	(102)
**Actinomycin D**	Pancreatic cancer	Down-regulating c-FLIP in HPAF, Panc1, Miapaca2, Bxpc3, Panc89, SW979, and Aspc1 cells (*in vitro*)	(103)
**Actinomycin D**	NSCLC	Increased expression of DR5 and caspase activation (*in vitro* and *in vivo*)	(104)
**PPARy ligands**	Prostate cancer	Down-regulating c-FLIP in prostate cancer, PPC-1 and LNCaP, ovarian cancer, OVCAR-3, and SK-OV-3 cells (*in vitro*)	(105)
	Ovarian cancer		
**YM155**	Cervical cancer	Downregulation of cFLIP and surviving in HeLa cells (*in vitro*)	(106)
**YM155**	Breast cancer	The p38 MAPK- and CHOP-mediated DR5 up-regulation (*in vitro* and *in vivo*)	(107)
**YM155**	RCC	Down-regulation of Mcl-1 and NF-κB-mediated down-regulation of c-FLIP expression in Caki cells (*in vitro*)	(108)
**Triciribine**	Prostate cancer	Dow-regulating Akt pathway in PC-3 and LNCaP cells (*in vitro*)	(109)
**PBOX**	Leukemia	Up-regulation of DR5, reduction of cellular mitochondrial potential, activation of the caspase cascade, and down-regulation of PI3K/Akt, c-FLIP, Mcl-1, and IAP survival pathways (*in vitro*)	(110)
**SNX-2112**	Cervical cancers	Inducing ROS-mediated JNK-p53-autophagy-DR5 pathway, and down-regulating Bcl-2, Bcl-xL, and c-FLIP in HeLa cells (*in vitro*)	(111)
**Progesterone**	Ovarian cancers	Down-regulating c-FLIP in OVCA 420, OVCA 429, and OVCA 433 cells (*in vitro*)	(112)
**ABT-737**	Various cancers	Up-regulation of DR5 (*in vitro*)	(113)
**ZFL**	RCC	Downregulation of Bcl-2 and Cbl-mediated c-FLIP by ROS-mediated p53 expression in Caki cells (*in vitro*)	(114)
**Bortezomib**	MM	Down-regulating c-FLIP (*in vitro*)	(115)
	RCC		
**c-Met inhibitor**	Liposarcoma	Up-regulation of DR5 in patient-derived cells (PDCs) (*in vitro*)	(116)
**Vemurafenib**	ATC	Dow-regulating Akt pathway in C643, CAL62, HTh7 cells (*in vitro*)	(117)
**Birinapant**	Breast cancers	Down-regulating c-FLIP in MDA-MB-453 cell (*in vitro*)	(118)
**ABC294640**	NSCLC	Up-regulating DR4/5, and inducing caspase-3, -8 expression (*in vitro*)	(119)
**Docetaxel**	Prostate cancers	Inducing ER stress in DU145 and PC3 cells (*in vitro*)	(120)
**Cabazitaxel**			

TRAIL, Tumor necrosis factor–related apoptosis-inducing ligand; DR4/5, Death receptor 4/5; PARP, Poly(ADP-ribose) Polymerase; JNK, Jun N-terminal kinase; FADD, Fas -associated death domain protein; HDAC4, Histone deacetylase 4; c-FLIP, Cellular FLICE (FADD-like IL-1β-converting enzyme)-inhibitory protein; ERK1/2, Extracellular signal–regulated protein kinase 1/2; 4E-BP1, Eukaryotic translation initiation factor 4E-binding protein 1; CHOP, C/EBP homologous protein; XIAP, X-linked inhibitor of apoptosis protein; NF-κB, Nuclear factor kappa B; Bcl-2, B-cell lymphoma-2; Bcl-xL, B-cell lymphoma-extra large; PI3K/AKT, Phosphatidylinositol 3-kinase; Bax, Bcl-2 associated X; Mcl-1, Myeloid-cell leukemia 1; Cbl, Casitas B-lineage lymphoma; ROS, Reactive oxygen species; (ER) stress, Endoplasmic reticulum; MM, Multiple myeloma; HNC, Head and neck cancer; RCC, Renal cell carcinoma; ATC, Anaplastic thyroid cancer; HCC, Hepatocellular carcinoma; NSCLC, Non-small cell lung cancer; SAHA, Suberoylanilide hydroxamic acid; VPA, Valporate; 5-FU, Fluorouracil; YM155, Sepantronium bromide; PBOX, Pyrrolo-1,5-benzoxazepine.

RETRACTED

### Natural Products

In addition to the synthetic agents, natural products have shown remarkable competence to improve apoptosis in resistant cell lines and also in tumor-bearing mice. In this regard, upregulation of DRs in association with affecting pro-and anti-apoptotic proteins in tumors is responsible for sensitizing TRAIL-resistant cells to TRAIL following combination treatment with natural products (121). For instance, toosendanin (TSN) as a triterpenoid derivative could render human primary NSCLC cells or NSCLC cell lines susceptible to TRAIL-induce apoptosis *in vitro* and *in vivo* largely through DR5 up-regulating and activation of CCAAT/enhancer-binding proteins (C/EBP) involved in endoplasmic reticulum (ER) stress response (122). Also, another natural product Taraxacum officinale F.H. Wigg (TO) currently has been suggested as a novel TRAIL sensitizer, as shown in human liver cell line Huh7 by suppressing MAP kinase kinase 7 (MKK7)‐TOR signaling pathway regulator‐like (TIPRL) interaction and subsequent activation of MKK7‐JNK phosphorylation (123). Further, TRAIL plus cantharidin, a type of terpenoid mainly extracted from the blister beetles (Mylabris genus), resulted in significant apoptosis in TRAIL−resistant prostate cancer DU145 cells. Importantly, observations signified that downregulation of c−FLIP accompanying with upregulation of DR5, supported TRAIL−induced apoptosis by initiating the autophagy flux (124).

Among a myriad of natural products, flavonoids have been proposed as one of the most powerful ingredients which can facilitate TRAIL-mediated apoptosis in resistant tumors. In this regard, some evidence has shown that flavonoid apigenin and genistein evidently increased TRAIL-mediated cytotoxicity against cervical cancer HeLa cells, while kaempferol and quercetin elicited no desired effects (125). Also, flavonoid resveratrol isolated from Artocarpus communis exerted caspase-dependent apoptosis, improved caspase 3/7 activity, and reinforced the protein levels of p53 and DR5 in gastric cancer cell lines, AGS, following combination therapy with TRAIL (126). Besides, flavonoid apigenin could connect and block adenine nucleotide translocase-2 (ANT2) activation, which led to inducing TRAIL-mediated apoptosis by DR5 up-regulating in TRAIL-resistance tumor cells, and thereby implying that ANT2 inhibitors may contribute to TRAIL therapy due to the ANT2 negative effects on DR5 expression on tumor cells (127). Moreover, flavonoid kaempferol elevated cytotoxic effects of the TRAIL on human ovarian cancer cells OVCAR-3 and SKOV-3 cells mainly mediated by up-regulation of DR4/5, CHOP, JNK, ERK1/2, p38, and down-regulating Bcl-2, Bcl-Xl, survivin, XIAP, and also c-FLIP. Silencing CHOP and DR5 evidenced the contribution of CHOP in DR5 up-regulation and also the involvement of DR5 in kaempferol-enhanced TRAIL-induced apoptosis (3). Similarly, DR5 up-regulation in a transcription factor CHOP-dependent manner was shown during tumor cell treatment with TRAIL and capsaicin (128), and also silibinin (129) in glioma cells. Also, our studies with leukemia MOLT-4 cells demonstrated that kaempferol could act as a sensitizer leading to sustained TRAIL-mediated apoptosis in MOLT-4 cells by up-regulating DR4/5 expression, reducing the expression of the NF‐κB subunit, and also down-regulating c-FLIP, X-IAP, and cIAP1 expression (130). Also, in another study, we showed that similar mechanisms are involved in stimulating TRAIL-mediated apoptosis in leukemia KG-1 cells following combination treatment with TRAIL and flavonoid quercetin (17). Similarly, apigenin, kaempferid, galangin, and caffeic acid phenylethyl ester (CAPE) in combination with TRAIL exerted remarkable cytotoxicity against prostate cancer cell lines, LNCaP (131). Besides, it has been shown that modifying WNT/β‐catenin and JAK‐STAT pathways, and also inhibiting the NF-κB pathway, may be involved in TRAIL-induced apoptosis in NSCLC xenografts following treatment with apigenin plus TRAIL (5). On the other hand, gingerol as a phenol phytochemical ingredient found in fresh ginger could reduce survivin, c-FLIP, Bcl-2, and XIAP expression, and restore pro-apoptotic protein Bax and tBid by producing reactive oxygen species (ROS), enabling TRAIL-mediated apoptosis in TRAIL-resistant glioblastoma cells (132).

RETRACTED

A list of the natural products which recently have been applied to sensitize tumor cells to TRAIL-induced apoptosis has been cited in **Table 2**.

**Table 2:** Combination therapy with natural products and TRAIL for improving TRAIL-mediated apoptosis in TRAIL-resistance cells.

Agent	Cancer	Mechanisms	Ref
**Piperine**	Breast cancer	Inhibition of survivin and p65 phosphorylation (*in vitro* and *in vivo*)	(133)
**Chalcones**	Prostate cancer	Changes of mitochondrial membrane potential (ΔΨm) in LNCaP cells (*in vitro*)	(134, 135)
**Chalcones**	Cervical cancer	Enhancement of expression of DR5 in HeLa cells (*in vitro*)	(136)
**Withanolides**	Renal carcinoma	Increasing cFLIP degradation (*in vitro* and *in vivo*)	(137)
**EEP**	Prostate cancer	Disruption of ΔΨm in LNCaP cells (*in vitro*)	(138)
**Curcumin**	Prostate cancer	Inducing cleavage of procaspase-3, procaspase-8, and procaspase-9, truncation of Bid, and release of cytochrome c in LNCaP cells (*in vitro*)	(139, 140)
**Chrysin**	Colon cancer	Activation of caspase 8 in HCT-116 cells (*in vitro*)	(141)
**Chrysin**	Lung cancer	Mcl-1 downregulation by inhibiting STAT3 phosphorylation in A549 and HeLa (*in vitro*)	(142)
	Cervical cancer		
**Embelin**	Pancreatic cancer	Down-regulation of XIAP and c-FLIP in TRAIL-resistant PC-1 cells (*in vitro*)	(143)
**Embelin**	Glioma	Activation of caspases 3, 7, 8, 9 and inhibition of c-FLIP (*in vitro*)	(144)
**Resveratrol**	Neuroblastoma	Down-regulation of Bcl-2 and survivin in SHEP cells (*in vitro*)	(145)
**Resveratrol**	Prostate cancer	Down-regulation of Bcl-2, Bcl-xL, and survivin and up-regulation of the expression of Bax, Bak, PUMA, Noxa, and Bim, and DR4/5 in prostate cancer PC-3 and DU-145 cells	(146)
**Resveratrol**	Melanoma	Attenuation of the STAT3 and NF-κB activation, activating JNK and down-regulating c-FLIP and Bcl-xL (*in vitro*)	(147)
**Berberine**	Prostate cancer	Upregulation of DR5 (*in vitro*)	(148)
	Liver cancer		
**Kaempferol**	Ovarian cancer	Targeting JNK/ERK-CHOP pathway and up-Regulation of Death Receptors 4 and 5 in OVCAR-3 and SKOV-3 cells (*in vitro*)	(3)
**Kaempferol**	Leukemia	Upregulation of DR4/5 and down-regulation of c-FLIP, XIAP, c-IAP in MOLT-4 cells (*in vitro*)	(130)
**Quercetin**	Leukemia	Upregulation of DR4/5 and inhibition of NF-κB in KG-1 cells (*in vitro*)	(17)
**Quercetin**	Liver cancer	Inhibition of NF-κB activation (*in vitro* and *in vivo*)	(149)
**Quercetin**	Pancreatic cancer	Down-regulation of c-FLIP (*in vitro*)	(150)
**Icariin**	Colon cancer	ROS-ERK-CHOP-mediated upregulation of DR5 and DR4 in HCT-116 cells (*in vitro*)	(151)
**Azadirone**	Colon cancer	ROS-ERK-CHOP-mediated up-regulation of DR5 and DR4 signaling and down-regulation of the Bcl-2, Bcl-xL, c-IAP-1, c-IAP-2, XIAP, survivin, Mcl-1 (*in vitro*)	(152)
**Irigenin**	Gastric cancer	Up-regulation of cleaved caspase-8, -9, and -3 and PARP and down-regulation of c-FLIP, Bcl-2, and survivin (*in vitro* and *in vivo*)	(153)
**Galangin**	Vrious cancer	Inducing TRAIL/caspase-3/AMPK signaling pathway (*in vitro*)	(154)
**Pterostilbene**	Breast cancer	Downregulation of c-FLIP, Bcl-xL, Bcl-2, survivin, and XIAP, and up-regulation of DR4 and DR5 through ROS-ERK-CHOP in TNMC cells (*in vitro*)	(155)
**Auriculasin**	Prostate cancer	Up-regulation of DR4/5, Bax, PARP, AIF, endonuclease G, and cytochrome c, and down-regulation of phosphorylation of AKT and mTOR, PI3K in RC-58T/h/SA#4 primary prostate cancer cells (*in vitro*)	(156)
**Kurarinone**	Gastric cancer	Downregulation of Mcl-1 and c-FLIP *via* inhibiting STAT3 signaling in SGC7901 cells (*in vitro*)	(157)
**Delphinidin**	Prostate cancer	Inducing DR5 and caspase-mediated HDAC3 cleavage (*in vitro*)	(158)
**Luteolin**	Lung cancers	Increasing DR5 expression and Drp1-mediates mitochondrial fission in A549 and H1975 cells (*in vitro*)	(159)
**Apigenin**	Prostate cancer	Up-regulation of DR5 and binding and inhibiting ANT2 in DU145 cells (*in vitro*)	(127)
**Genistein**	Lung cancer	increased LC3-II, p62, activated caspase-3, and activated caspase-8 accumulation in A549 cells (*in vitro*)	(160)
**Celastrol**	Lung cancer	Modifying of ROS and ΔΨm and up-regulation of active caspase 3 and 8 (*in vitro*)	(161)
**Biochanin-A**	Prostate cancer	Inhibition of transcription factor NF-κB(p65) activity, promotion of DR5 expression, and disruption of ΔΨm in LNCaP and DU145 cells (*in vitro*)	(162)
**Fisetin**	Prostate cancer	Upregulation of DR4, caspase 3, 8 and downregulation of NF-κB activation (*in vitro*)	(163)
**Liquiritin**	Gastric cancer	ROS generation (*in vitro* and *in vivo*)	(164)
**Codium extracts**	Colon cancer	Degradation of c-FLIP (*in vitro*)	(165)
**Ampelopsin**	EBV+ cancers	Upregulation of TRAIL/DR5 and activation of p38 signaling (*in vitro*)	(166)
**Xanthohumol**	Neuroblastoma	Up-regulation of DR5 (*in vitro* and *in vivo*)	(167)
**Luteolin**	Pancreatic cancer	Affecting miR-301-3p/caspase-8 axis in PANC-1 cells (*in vitro*)	(168)

TRAIL, Tumor necrosis factor–related apoptosis-inducing ligand; DR4/5, Death receptor 4/5; STAT3, Signal transducer and activator of transcription 3; JNK, Jun N-terminal kinase; FADD, FAS-associated death domain protein; c-FLIP, Cellular FLICE (FADD-like IL-1β-converting enzyme)-inhibitory protein; ERK1/2, Extracellular signal–regulated protein kinase 1/2; CHOP, C/EBP homologous protein; XIAP, X-linked inhibitor of apoptosis protein; NF-κB, Nuclear factor kappa B; Bcl-2, B-cell lymphoma-2; Bcl-xL, B-cell lymphoma-extra large; PI3K)/AKT, Phosphatidylinositol 3-kinase; Mcl-1, Myeloid-cell leukemia 1; ROS, Reactive oxygen species; ER stress, Endoplasmic reticulum; Bax, Bcl-2 associated X; Bak, Bcl-2 homologous antagonist/killer; Bid, BH3-interacting domain death agonist; PUMA, P53 upregulated modulator of apoptosis; Noxa, Phorbol-12-myristate-13-acetate-induced protein 1; c-IAP, Cellular inhibitor of apoptosis; PARPs, Poly (ADP-ribose) polymerases; AMPK, AMP-activated protein kinase; AIF, Apoptosis inducing factor; DRP1, Dynamin-related protein 1; ANT2, Adenine nucleotide translocator 2; mTOR, Mechanistic target of rapamycin; LC3, Microtubule-associated protein 1A/1B-light chain 3; EEP, Ethanolic extract of propolis.

RETRACTED

## Trail Delivery Using NPs

Nanoparticles (NPs) have been applied as an operational delivery carrier for s diverse types of anticancer drugs. The molecular self-assembly of active proteins has attracted huge attention for nanomaterials advancement. Protein-based NPs established by TRAIL and diphenylalanine (FF) (TRAIL-FF) by molecular self-assembly could be constructed by adjusting the concentration and the two ingredients ratio. Established NPs could induce apoptosis signaling pathways in human breast cancer MCF-7 cells and lung H460 cells due to a particular interface between TRAIL and death receptors, suggesting that the application of protein-based functional biomaterials is a rational strategy for treating human cancers (169). Further, magnetic ferric oxide NP-conjugated TRAIL (NP-TRAIL) could stimulate apoptosis, reduce tumor volume, and improve the overall survival rate in U251 cell-derived xenografts. Moreover, combined treatment with NP-TRAIL and γ-radiation or bortezomib could sensitize TRAIL-resistant glioblastoma cancer stem cells (CSCs) to NP-TRAIL. Thereby, these findings offer proof of the idea that conjugation of TRAIL to NP can improve its apoptotic functions both *in vitro* and *in vivo* (170). Similarly, artificial lipid NPs coated with TRAIL powerfully ameliorated TRAIL cytotoxic activities in chemoresistant hematological cancer cells and NSCLC, possibly mediated by up-regulating caspase-8 and caspase-3 activation (171). Besides, TRAIL-coated gold nanoparticles (TRAIL-AuNPs) robustly induced apoptosis in NSCLC by inducing mitochondrial fragmentation in tumor cells along with a marked promotion in mitochondrial recruitment of dynamin-related protein 1 (Drp1), inducing mitochondrial deficits, and supporting the autophagy process (172). On the other hand, TRAIL and curcumin (Cur)-coated NPs (TRAIL-Cur-NPs) resulted in boosted cellular uptake, cytotoxicity, and apoptosis-inducing influences on HCT116 colon cancer cells. More importantly, TRAIL-Cur-NPs showed remarkable anticancer *in vivo* effects without noticeable toxicity, which was mostly because of the high tumor targeting and synergistic impacts of TRAIL and Cur. Analysis indicated that upregulation of DR4 and DR5 on tumor cells stimulated by Cur was reliable for anti-tumor effects elicited by constructed NPs, suggesting that co-delivery of NPs may serve notable merits for cancer therapy (173). Moreover, Min et al. found that paclitaxel (PTX)-bound albumin NPs with embedded TRAIL (TRAIL/PTX HSA-NP) may be an effective option for treating pancreatic cancer. They showed that TRAIL/PTX HSA-NPs could stimulate more substantial apoptotic activity than plain PTX HSA-NP in pancreatic Mia Paca-2 cells *in vitro* and also in Mia Paca-2 cell-xenografted mice (174). Likewise, TRAIL/doxorubicin (Dox) HSA-NPs inhibited tumor growth in colon cancer HCT116 tumor-bearing BALB/c nu/nu mice. It was found that TRAIL/Dox HSA NPs infiltrated intensely into tumor masses in an HCT116 spheroid model and localized in the tumor area upon systemic injection (175). Furthermore, TRAIL-iron oxide NPs induced ROS-mediated JNK activation, which in turn, could support DR5 up-regulation, and subsequently promoted antitumor efficacy of TRAIL in TRAIL-resistant colon cancer HT-29, intermediately resistant SW-480 and sensitive HCT-116 cells, *in vitro*. TRAIL-iron oxide NPs also blocked tumor growth and prolonged the survival rate of xenografts compared with control and TRAIL monotherapy (32). As well, TRAIL delivery using polyethyleneimine (PEI)-poly[(1,6-hexanediol)-diacrylate-β-5-hydroxyamylamine] (PBAE) in TNBC (176), silver NPs (AgNPs) in glioblastoma (177), TPGS-b-(PCL-ran-PGA)/PEI NPs in cervical cancer (178), neutrophil membrane (NM)-based NPs in various cancers (179), and artificial lipid NPs in colon cancer (180), leukemia (181), sarcoma (182), and also TNBC (30) has been suggested as authentically and operational therapeutic approach.

RETRACTED

## Trail Delivery Using MSCs

It has been recently hypothesized that human MSCs engineered to generate and deliver TRAIL can infiltrate to and eliminate tumor cells in tumor models (**Table 3**). Accordingly, human MSCs transduced with TRAIL-induced apoptosis in lung cancer A549 cells, breast cancer MDAMB231 cells, squamous cancer H357 cells, and cervical cancer HeLa cells in co-culture experiments. As well, subcutaneous xenograft tests evidenced that directly transferred TRAIL-expressing MSCs could potently delay tumor growth (189). Also, TRAIL-expressing MSCs migrated to and reduced tumor burden in squamous H357 cell and lung A549 cell xenograft models. Correspondingly, engineered MSCs stimulated tumor cell apoptosis, and concomitantly decreased colony formation of the squamous and adenocarcinoma lung cancer cells (188). There is other proof signifying that TRAIL-expressing MSCs engineered by reconstituted high-density lipoprotein (rHDL) nanovector is an effective strategy for the treatment of pulmonary melanoma metastasis-targeting therapy. Observations have proposed that genetically engineered MSCs could strongly target B16F10 cells, thus making a substantial apoptosis-inducing impact on aggressive melanoma *in vitro* and *in vivo* (206). Other reports have proven that interferon (IFN)-β and TRAIL-expressing adipose tissue-derived MSCs (AT-MSCs) induced significant apoptosis in human lung cancer cell line H460 in co-culture experiment, and also reduced tumor burden in H460-derived cancer animal models. As well, it has been found that serum deprivation during cell culture triggered the expression of IFN-β and TRAIL by engineered AT-MSCs (207).

**Table 3:** MSCs-based delivery of TRAIL in human tumor cells.

TRAIL form	Cancer	Main result	Ref
**Soluble (s)**	Glioblastoma	Paclitaxel priming the of MSCs-TRAIL promoted antitumor functions of their secretome in CFPAC-1 and U87-MG cells (*in vitro*)	(183)
	Pancreatic cancer		
**Soluble**	Neuroblastoma	MSCs-TRAIL-induced apoptosis in neuroblastoma cells (*in vitro* and *in vivo*)	(184)
**Recombinant**	NSCLC	MSCs-TRAIL resulted in significant tumor cell inhibition in NSCLC-derived cancer stem cells (*in vitro*)	(185)
**Recombinant**	Breast	MSCs-TRAIL-induced cell death in a resistant type of breast cancer cells, MCF-7 (*in vitro*)	(186)
**Soluble** **Full Length (FL)**	Prostate cancer	MSC-sTRAIL showed more prominent anti-tumor effects than MSC-FL-TRAIL when used combined with AKT inhibitors in LNCaP, C4-2B, and PC3 cells (*in vitro*)	(187)
**Recombinant**	SCC	MSCs-TRAIL-induced apoptosis in H357 and A549 cells (*in vitro*)	(188)
	Lung cancer		
**Soluble**	Lung cancer	MSCs-TRAIL systemic injection into mice models resulted in a significant reduction in metastatic tumor burden with frequent eradication of metastases	(189)
	SCC		
	Breast cancer		
	Cervical cancer		
**Soluble**	Pancreatic cancer	MSCs-TRAIL and their secretome stimulated apoptosis in PANC1, HP62, ASPC1, TRM6, and BXPC3 cells (*in vitro*)	(190)
**Full Length**	Esophageal cancer	MSCs-TRAIL supported the inhibition of the proliferation and induced apoptosis in Eca-109 cells (*in vitro*)	(191)
**Full Length**	Breast cancer	MSCs-TRAIL systemic injection led to the reduced tumor burden in mice models	(192)
**Full Length**	Multiple myeloma	MSCs-TRAIL systemic injection resulted in decreased the tumor burden by specific induction of apoptosis in multiple myeloma cells as showed by caspase-3 activation in mice models	(193)
**Recombinant**	Lung cancer	MSCs-TRAIL systemic injection supported tumor growth inhibition in A549 xenograft mouse model	(194)
**Soluble**	Liver cancer	MSCs-TRAIL secretome led to the apoptosis induction in HepG2 cells (*in vitro*)	(195)
**Recombinant**	Multiple myeloma	MSCs-TRAIL in combination with bortezomib significantly stimulated myeloma cell apoptosis by caspase-8 activation (*in vitro*)	(196)
**Soluble**	Liver cancer	MSCs-TRAIL subcutaneous injection inhibited tumor growth and significantly increased survival in mice models mediate by up-regulating caspase 3 activation	(197)
**Recombinant**	NSCLC	MSCs-TRAIL administration caused a reduction in tumor size, tumor weight, and circulating tumor cells in the xenograft model	(198)
**Recombinant**	Glioblastoma	MSCs-TRAIL-induced apoptosis in C6 cells (*in vitro*)	(199)
**Recombinant**	Glioma	MSCs-TRAIL administration resulted in reduced tumor burden in glioma Fischer 344 rats	(200)
**Recombinant**	Mesothelioma	MSCs-TRAIL supported a reduction in malignant pleural mesothelioma tumor growth by an improvement in tumor cell apoptosis in xenograft models	(201)
**Soluble**	Various tumors	MSCs-FL-TRAIL showed superiority over MSCs-sTRAIL in terms of inducing anti-tumor effects in lung cancer lines, malignant pleural mesothelioma lines, colon cancer lines, renal cancer lines, oral squamous cell carcinoma line, and breast adenocarcinoma line (*in vitro*)	(202)
**Full Length**			
**Full Length**	Glioma	MSCs-TRAIL caused potent induction of apoptosis in gliomas cells leading to the reduced tumor burden in xenograft models	(203)
**Soluble**	Glioma	MSCs-TRAIL intratumoral injection supported inhibited tumor growth and prolonged the survival of glioma-bearing mice	(204)
**Soluble**	RCC	Complete regression of metastatic RCC by multiple infusion of MSCs expressing dodecameric TRAIL and HSV-TK into tumor-bearing mice	(205)

TRAIL, Tumor necrosis factor-related apoptosis-inducing ligand; MSCs, Mesenchymal stem/stromal cells; NSCLC, Non-small cell lung cancer; SCC, Squamous cell carcinoma; RCC, Renal cell carcinoma; HSV-TK, Herpes simplex virus-thymidine kinase.

RETRACTED

Combined treatment with TRAIL-expressing human MSCs and compound C, an AMP-activated protein kinase (AMPK inhibitor), resulted in remarkable anti-tumor effects on glioma cells *in vitro* and in *in vivo* models. Indeed, TRAIL-expressing MSCs plus compound C increased apoptosis by improving the expression of Bax accompanied by attenuating anti-apoptotic proteins c-FLIP, XIAP, and Bcl-2 in glioma; on the other hand, intervention promoted caspase-3 cleavage and apoptotic cells in a murine glioma model (208). Similarly, MSCs engineered to express TRAIL led to the death of classic and primary neuroblastoma cell lines *in vitro*. Although these TRAIL-engineered MSCs infiltrated into tumor tissue *in vivo*, they did not significantly modify neuroblastoma progress in murine models, indicating that MSCs could be applied to deliver therapeutic agents in neuroblastoma patients, whereas more effective biopharmaceuticals should be utilized instead of TRAIL (184). In another study, in addition to the preservation of their multipotent characteristic, TRAIL expressing MSCs co-cultured with CD133-positive CSCs facilitated a robust reduction in CSCs proliferation and triggered cancer cells apoptosis *in vitro* mainly inspired by stimulating the apoptosis intrinsic pathway. Molecular analysis demonstrated that adjusting the expression of NF-κB1, BAG cochaperone 3 (BAG3), Mcl-1, growth arrest, and DNA damage-inducible alpha (GADD45A), and harakiri (HRK) was responsible for achieved anti-tumor effects exerted by MSCs-TRAIL in CSCs (185). Similarly, TRAIL-expressing AT-MSCs was found to alleviate colon cancer by stimulating the apoptosis of CD133-positive CSCs and declining the M2 macrophage frequency (209). Importantly, other studies have shown that exosomes (Exos)-derived from TRAIL-expressing MSCs reduced tumor weight in tumor-bearing mice, indicating that MSC-derived Exo-TRAIL has a prospective ability for cancer therapy (210).

RETRACTED

## Trail-R Agonistic Monoclonal Antibody

Regardless of TRAIL interaction, agonistic antibodies targeting TRAIL-receptors can specifically stimulate apoptosis in tumor cells (211). For instance, a human agonistic TRAIL-R1 mAb, HGS-ETR1, established specific communication with the TRAIL-R1 receptor (DR4). HGS-ETR1 could decrease the viability of various types of tumor cells *in vitro*, and simulated activation of caspase-8, -9, -3, Bid, and cleavage of PARP, indicating that stimulation of DR4 alone is adequate to trigger both extrinsic and intrinsic apoptotic pathways. As well, combined treatment with HGS-ETR1 and chemotherapeutic agents, topotecan, 5-FU, and irinotecan caused restored anti-tumor function against colon cancer xenograft models (212). Moreover, a novel anti-human DR5 monoclonal antibody, TRA-8, could trigger apoptosis in HCC cells both *in vitro* and *in vivo*, while it has no cytotoxicity against normal hepatocytes (213). Also, the combination of cisplatin with mapatumumab, an agonistic mAb directed against DR4, or lexatumumab, an agonistic mAb directed against DR5, synergistically suppressed the cell proliferation and improved apoptotic death in malignant pleural mesothelioma (MPM) cell lines (214). Besides, Piao et al. showed that constructed mAbs to DR4 (TR1- IgMs) using ISAAC technology activated the caspase cascade and stimulated strong apoptosis in human tumor cell lines, such as breast cancer and lung adenocarcinoma cells, and also in the xenograft model (215).

In phase I and also in phase II clinical trials, mapatumumab has demonstrated a remarkable safety profile and, resulted in complete or partial clinical responses when injected as monotherapy in patients suffering from follicular NHL (216). Mapatumumab was shown to be well tolerated up to 20 mg/kg daily and its potent therapeutic effects has been investigated for treatment of NSCLC, multiple myeloma, NHL, and HCC (216, 217). Currently, a phase II multicenter study on 38 patients suffering from CRC verified the safety but not significant efficacy of the mapatumumab therapy (218).

The therapeutic benefits of combination therapies with mapatumumab were evaluated in several malignancies. Most of the combinations, including mapatumumab with paclitaxel, gemcitabine, carboplatin or bortezomib have not caused desired outcomes (219). Nonetheless, evaluation of the efficacy and safety of mapatumumab in combination with sorafenib in 101 patients with HCC revealed that intervention led to no significant beneficial effects on enrolled patients (220).

RETRACTED

Among the TRAIL-R2 agonistic antibodies, lexatumumab, drozitumab, DS-8273a, and LBY-135, have completed the phase I clinical trials. Further, tigatuzumab and conatumumab entered the phase II of clinical testing (217). Investigation of the possible anti-tumor effects of the agonistic antibody (DS-8273a) on 16 patients with advanced cancers evidenced that DS-8273a therapy resulted in the decrease of myeloid-derived suppressor cells (MDSC) in 50% of the patients, supporting DS-8273a utility in combination immunotherapy of cancer (221). However, in advanced NSCLC patients, tigatuzumab had no positive effect on the efficacy of carboplatin/paclitaxel (222). Besides, in metastatic pancreatic adenocarcinoma patients, conatumumab therapy led to the significant but not remarkable improvement in the 6-month survival rate as compared to the placebo (223).

## Conclusion

During the last decades, exploration for innovative cancer therapeutics has concentrated on the aim of advancing specific, targeted, and less toxic molecules/drugs for cancer therapy (224). In this regard, TRAIL as a capable chemotherapeutic ingredient has attracted considerable attention; however, TRAIL therapy has faced some limitations in the clinical setting. Although the exact mechanisms contributing to the escape from TRAIL-induced apoptosis and progress of resistance to TRAIL in tumor cells has not yet been found completely, it seems that down-regulating pro-apoptotic proteins and DR4/5, concomitant with up-regulating anti-apoptotic proteins along with activating some signaling axis plays an influential role in this regard (225, 226). Nonetheless, it is still not elucidated whether the cellular procedures alone or in combination can stimulate resistance to TRAIL. As described, pre-clinical reports have ideated that combination therapy with a natural product or synthetic agents can make TRAIL-resistant cells susceptible to TRAIL-induced apoptosis (227, 228). Moreover, TRAIL-targeted delivery using human MSCs and also NPs has been considered an effective strategy for overcoming resistance to TRAIL (229, 230). In sum, we suggest that operational therapeutic modification of TRAIL resistance principally need to focus on the progression of approach for improving the half-life of TRAIL, recognition of appropriate biomarkers by pre-selection of patients that show suitable response to TRAIL/agonist antibody therapy, advancement of novel synergistic combinations with TRAIL and blocker of cell stress response proteins, and finally detection of novel TRAIL sensitizers from FDA approved drug libraries.

RETRACTED

## Author Contributions

All authors contributed to the conception and the main idea of the work. ER, HR, WA, DB, MY, WS, AH, and FM drafted the main text, figures, and tables. MJ supervised the work and provided the comments and additional scientific information. ER and FM reviewed and revised the text. All authors contributed to the article and approved the submitted version.

## Conflict of Interest

The authors declare that the research was conducted in the absence of any commercial or financial relationships that could be construed as a potential conflict of interest.

## Publisher’s Note

All claims expressed in this article are solely those of the authors and do not necessarily represent those of their affiliated organizations, or those of the publisher, the editors and the reviewers. Any product that may be evaluated in this article, or claim that may be made by its manufacturer, is not guaranteed or endorsed by the publisher.
